# Comparing Soil Erosion Rates on Terraced and Sloping Cultivated Land in Palestine Using FRN ^137^Cs Trace

**DOI:** 10.1155/2022/2933661

**Published:** 2022-09-30

**Authors:** Orwa Houshia, Moncef Benmansour, Lionel Mabit, Emil Fulajtár, Saber Abu-Jabal, Ismail Hroub, Rafat Odeh

**Affiliations:** ^1^Department of Chemistry, Arab American University, Jenin, State of Palestine; ^2^Centre National de L'Energie des Sciences et des Technique Nucleaires (CNESTEN), Division of Water, Soil and Climate, Rabat, Morocco; ^3^Soil and Water Management and Crop Nutrition Laboratory, The International Atomic Energy Agency (IAEA), Seibersdorf, Vienna, Austria; ^4^Soil and Water Management & Crop Nutrition Section, Joint FAO/IAEA Division of Nuclear Techniques, Food and Agriculture, International Atomic Energy Agency, Vienna, Austria; ^5^Department of Chemistry, An-Najah National University, Nablus, State of Palestine; ^6^Radiation Protection & Detection Unit, Ministry of Health Qadoora Street Ramallah, Ramallah, State of Palestine

## Abstract

Soil erosion is a serious problem in Palestine. It is enhanced mainly by poor farming practices used in upland agricultural areas occupying the Central Highland of Palestine. The objective of this study is to assess the impact of terracing on soil erosion and deposition rates in the Al-Yamoun area (the Northern West Bank) using the fallout radionuclides cesium -137 (FRN ^137^Cs). The FRN ^137^Cs technique, which has proved its efficiency in estimating erosion rates over the last 50–60 years, was used for the first time in Palestine to measure rates of erosion and deposition. The activity of ^137^Cs was measured by gamma spectrometry using an HPGe detector. For the reference site, the ^137^Cs inventories ranged between 2499 and 4086 Bq/m2. The average value of the reference site is 3315 ± 410 Bq/m2, which corresponds to a coefficient of variance of 12%, suggesting that the reference site is well representative for estimating 137Cs fallout. This ^137^Cs amount is too high for bomb-derived fallout and indicates that a significant part of the deposition is from the Chernobyl accident. The ^137^Cs inventories at both studied sites (terrace site and foot slope site) are significantly lower than those of the reference site. For the terrace site, the inventories are found between 1707 and 2749 Bq/m2, while for the slope site they are between 1050 and 2617 Bq/m2. The lower ^137^Cs values at both studied sites than values at the reference site indicate that the entire areas of both study sites are eroded and no depositional activity occurs.

## 1. Introduction

Agriculture is an important cultural tradition vital to the economy of the West Bank, Palestine. Also, agriculture plays a vital role in the region's future. Palestinians are coping in creative ways [1] every day despite the challenges of establishing a livelihood or any sustainable economic activity based on agriculture. Whether the challenge lies in water scarcity, soil degradation [2], or blockade restrictions, Palestinian families implement innovative and collaborative approaches to living off the land [3]. However, the land suitable for agriculture in Palestine is shrinking due to soil erosion, land degradation, and water erosion, which in turn affect soil properties and functions [4–7] and cause the loss of soil, which is not renewable on the human timescale. Consequently, these factors represent a major threat to the soil and water resources the country needs to ensure sustainable agricultural production.

Within this context, and in order to provide a comprehensive assessment of the magnitude of these problems and to support the selection of effective soil conservation measures, quantitative data on the extent and rates of soil erosion under various agroecological conditions and land use systems were needed [8]. Integrated land and water management practices improve agricultural production and enhance soil productivity and its resilience against desertification and other impacts of climate change and variability. Radionuclide and stable isotopic techniques can be used to study soil erosion and land degradation problems [9]. Data on soil erosion acquired by conventional methods takes several years to obtain and is time consuming. Furthermore, it is labor-intensive, and these conventional methods do not provide for the spatial distribution of soil erosion. On the other hand, the 137Cs isotope tracer fills the deficits of the conventional methods and facilitates the investigation of soil erosion on a much better timescale, so there is no need for costly, labor-intensive long-term monitoring.

## 2. Methodology

### 2.1. Study Area

The study area is located in the Central Highland in the Jenin Province, which receives annual precipitation of about 300 mm (Figure 1). The sampling sites were selected to acquire soil samples within the Jenin Province. The reference site at an elevation of 293 m above sea level was covered with shrub vegetation and had a slope of about 2%. The other two sites were labeled Terrace Site, which at an elevation of 246 m above sea level, cultivated land on a terrace with a slope of 2%, and foot slope site, which at an elevation of 140 m above sea level, cultivated land on a foot slope that was not terraced and had a slope of 3%. The difference in slope inclination is very small, but the important difference is the slope length (field length), which is very short on the terrace (10–15 m) and several folds longer at the foot slope field (60 m).

### 2.2. Field Sampling

The sampling design is as follows:

#### 2.2.1. Reference Site

Grid samplingof 1.5 m (24 samples) (3 × 8), bulk samples, 30 m depth, and a distance between two points is of 1.5 m.

#### 2.2.2. Terrace site

Sampling along 3 transects containing 8 points in each transect (24 soil samples), bulk samples, 30 cm depth, and a distance of 1.5 m between two points.

#### 2.2.3. Foot slope site

Sampling along 3 transects containing 8 points in each transect (24 soil samples), bulk samples, 30 cm depth, and a distance of 1.5 m between two points.

## 3. Sample Preparation and ^137^Cs Analysis

Physical preparation of the soil samples was performed at the Palestine National Agricultural Center (NARC) including drying and light grinding. Then, samples were oven dried at 105 degrees Celsius, grinded, sieved (<2 mm), and homogenized. Radionuclide analysis of ^137^Cs was performed by gamma spectrometry using an HPGe detector (45 efficiencies) by the Centre National de l'Energie des Sciences et des Technique Nucleaires (CNESTEN), Morocco. Tennelec/Nucleus HPGe (184 cc) planar-type coaxial intrinsic germanium detector was used. The ^137^Cs activity was measured by its gamma emission at 662 keV. Background counts were made at regular intervals to ensure the maintenance of low background characteristics. Each soil sample was counted for 20000 s. The Cs inventory A (Bq·m^−2^) was calculated using the following equation:

(1) $$\begin{array}{c} A=\frac{CM}{S}, \end{array}$$

where C is the ^137^Cs activity concentration of the sample (in Bq·kg^−1^), *M* is the total dry mass of the collected soil core (in kg) and S is the cross-section of the sampling tube (in m^2^)

## 4. Results and Discussion

Numerous models were established to analyze soil erosion [10]. The main postulates and necessities of the ^137^Cs approaches have been reported in several papers [11]. The calculation of soil erosion and deposition rates at the undisturbed site is based on ^137^Cs inventories and the ^137^Cs depth distribution. Two methods are used. The simpler method considers the fixed ^137^Cs fallout input and stable ^137^Cs profile distribution. The depth distribution over the soil profile is mathematically described [12]. If this distribution is considered by a simple mathematical function, then the soil loss can be estimated by the proportion of the ^137^Cs reference value removed at the examined site [13]. This method is used for the Profile Distribution Model (PDM). A more widespread method takes into consideration the time-variant processes of: (1) the ^137^Cs fallout and (2) the gradual postdepositional redistribution of ^137^Cs within the soil profile, which is caused predominantly by bioturbation and several other processes. This approach is used by the Diffusion and Migration Model (DMM) [14]. The calculation of soil loss in cultivated land can be based on two theoretical concepts. The first one called, the proportional concept, is very simple and it presumes that the removal of soil and ^137^Cs are directly proportional. Models based on this concept are called the Proportional Model (PM). More complex approaches involve a mass balance concept, which considers the temporal dynamics of ^137^Cs inputs and outputs resulting in the time-variant concentration of ^137^Cs in soil [12]. These changes in concentration affect considerably the relation between the ^137^Cs loss and soil loss caused by erosion. The ^137^Cs concentration in soil is controlled by several processes [13, 15–17]. Most important are (1) time-variable 137Cs fallout, (2) radioactive decay of ^137^Cs (i.e., 30.17 years), (3) removal of freshly deposited ^137^Cs by erosion prior to its incorporation into the plough horizon by tillage, and (4) incorporation of subsoil material free of ^137^Cs or having low ^137^Cs content into the eroded ploughed horizon by tillage [18].

The Mass Balance Models (MBM) were developed in the mid-1980s. Different models use different approaches to handle the ^137^Cs time-variant concentration in soil and consider some but not all processes and factors controlling it [12, 19, 20]. Moreover, three Mass Balance Models that were initially developed by Walling and He [10] are used, e.g., Mass Balance Model 1 (MBM1), Mass Balance Model 2 (MBM2), and Mass Balance Model 3 (MBM3).

In order to convert inventories or areal activities (in Bq/m^2^) into soil erosion or deposition rates (in t/ha/yr), conversion models were used. First, the Proportional Model (PM) was used to have preliminary results about soil erosion, in accordance with equations (2), (3), and (4) obtained from references [12, 21].

The basic equation (2) of the Proportional Model [10] can, therefore, be represented as follows:

(2) $$\begin{array}{c} Y=10\frac{BdX}{100TP}, \end{array}$$

where *X* is the percentage reduction in total ^137^Cs inventory (defined as (A_ref_ -A)/A *∗* 100), *d* is the depth of the plough or cultivation layer (m), B is the bulk density of the soil (kg·m^−3^), *T* the time elapsed since the start of ^137^ Cs accumulation (yr), A_ref,_ represents the local reference inventory (Bq·m^−2^), and A is the total inventory measured at the sampling point (Bq m^−2^). P represents the particle size correction factor for erosion. This model does not require many parameters, but it is not realistic as he neglected some processes or phenomena related to ^137^Cs behavior and erosion processes in cultivated sites.

In addition, the Chernobyl contribution was not included when applying this model. In this case, Mass Balance Models were used (equation (3)) and, more specifically, the Mass Balance Model 2, which can describe suitably the real situation and therefore was also applied (equation (4)). It has to be noted that the file for the annual deposition of ^137^Cs was modified to take the Chernobyl contribution into account. The results given by both models for both sites 1 and 2 are reported in Table1 and Table 2.

(3) $$\begin{array}{c} Y=10dB\;{\left(1-\left[1-\frac{x}{100}\right]\right)}^{1/\left(t-1963\right)}, \end{array}$$

where *t* represents the time since 1963, B is the bulk density of the soil (kg·m^−3^), and *d* is the depth of the plough or cultivation layer (*m*). *X* is the percentage reduction in total 137 Cs inventory (defined as (A_ref_ -A)/A *∗* 100)

(4) $$\begin{array}{c} \frac{\text{d}A\left(t\right)}{\text{d}t}=\left(1-\Gamma \right)I\left(t\right)-\left(\lambda +P\frac{R}{d}\right)A\left(t\right), \end{array}$$

where A (t) = cumulative ^137^Cs activity per unit area (Bq/m^2^); *R* = erosion rate (kg/m^2^. yr) *d* = cumulative mass depth, representing the average plough depth (kg/m^−2^) *λ* = decay constant for ^137^Cs (yr^−1^); I (t) = annual ^137^Cs deposition flux (Bq/m^2^ yr); Γ = percentage of the freshly deposited ^137^Cs fallout removed by erosion before being mixed into the plough layer; *P* = particle size correction factor.

The inventories of the samples were calculated from the ^137^Cs concentration (in Bq/kg), the bulk density of the sample, and the depth of the core. An average bulk density was calculated for each type of site. There are about 1160 kg/m^3^, 1240 kg/m^3^, and 1190 kg/m^3^ for a reference site, site 1, and site 2, respectively.

The results of all inventories (Bq/m^2^) are given in Table 3. For the reference site, the inventories ranged between 2927 and 4086 Bq/m^2^. The average value of the reference site is 3315 ± 410 Bq/m^2^, which corresponds to a coefficient of variance of about 12%. This coefficient of variance can be considered as low, confirming the low variability and low disturbance of the selected reference site. The high inventory associated with the reference site suggests that the fallout ^137^Cs deposited in this region is the result of both old nuclear weapon tests conducted in the 1950s–1960s and the Chernobyl disaster that occurred in 1986. Taking into account the average rainfall in this region (Jenin Province) of about 300 mm, the inventory estimated by prediction using conversion models is about 897 Bq/m^2^. It means that the contribution of Chernobyl is about 2418 Bq/m^2^, which represents around 73% of the total reference inventory. Concerning study site 1 and site 2, the inventories are significantly lower than those of the reference site (see Table 1), especially for site 2, indicating that these sites are eroded.  Figure 2 shows the distribution of ^137^Cs inventory along 3 transects for each site and the mean reference inventory value. For site 1, inventories are found between 1707 and 2749 Bq/m^2^, while for the site 2, inventories are found between 1050 and 26117 Bq/m^2^. In comparison, all the inventories obtained are lower than the reference value (Figure 1), indicating that there is no depositional area at both sites.

As previously reported by Nouira et al. [19], the Proportional Model does not take into account the dilution of ^137^ Cs concentrations in the soil within the cultivated layer, resulting from the assimilation of soil from below the originally cultivated depth due to surface lowering by erosion; thus, the results obtained by this model in the present study likely underestimate the actual rates of soil loss. The Mass Balance approach that takes into account the effect of mixing the subsoil containing no ^137^Cs from below the plough depth into the plough layer gave higher values for soil loss rate, as is observed in some other reports [19, 22].

## 5. Conclusions

^137^Cs distribution at the sites confirmed that the ^137^Cs tracking procedure can be effectively used to assess soil erosion and deposition rates. The application of the ^137^Cs tracking system enabled us to quantify the extent of soil erosion in the Northern Palestine region. For the reference site, the inventories ranged between 2927 and 4086 Bq/m^2^. The average value of the reference site is 3315 ± 410 Bq/m^2^, which corresponds to a coefficient of variance of about 12%, suggesting that the fallout 137Cs deposited in this region is a result of both old nuclear weapon tests conducted in 1950s–1960s and the Chernobyl disaster that occurred in 1986.

Finally, the ^137^ Cs tracking technique is a useful erosion model for the Northern Palestine region. This data can be used to refine erosion control guidelines influencing the selection of a vast array of management practices by an agricultural producer, such as tillage, fertilizer application, crop rotation, plant population, and structures. Thus, the future work, which will be carried out in phase–II of the project, highly recommends the selection of more locations in Gaza and the West Bank in order to generate a soil erosion map of Palestine. This result will also be presented to legislators and decision makers within the government to implement appropriate soil erosion solutions.

## Figures and Tables

**Figure 1:** Location of the study area. The inset picture is an aerial view of the actual locations.

**Figure 2:** ^137^Cs inventories (Bq/m^2^) along 3 transects associated with site 1 (a) and site 2 (b).

**Table 1:** Soil erosion rates in t/ha/yr associated with site 1 for different points of the transects using the Proportional Model (PM) and Mass Balance Model 2 (MBM2).

Foot slope site 1						
Distance from the top (m)	PM			MBM2		
	T1	T2	T3	T1	T2	T3
0	9.6	18.8	8.7	10.9	26.7	9.6
1.5	11.1	7.1	9.5	13.0	7.7	10.7
3	7.4	15.6	7.7	8.1	20.3	8.4
4.5	11.5	8.1	7.3	13.6	8.9	7.9
6	17.4	8.1	9.3	23.9	8.9	10.5
7.5	16.7	5.4	8.2	22.4	5.7	9.0
9	5.9	10.0	6.6	6.2	11.4	7.1
10.5	11.1	7.2	9.5	12.9	7.8	10.7

**Table 2:** Soil erosion rates t/ha/yr associated with site 2 for different points of the transects using the Proportional Model (PM) and Mass Balance Model 2 (MBM2).

Terraced site 2						
Distance from the top (m)	PM			MBM2		
	T1	T2	T3	T1	T2	T3
0	22.9	23.5	10.0	40.0	42.4	12.0
1.5	22.3	16.5	9.4	38.2	23.3	11.2
3	21.8	10.9	12.0	36.6	13.3	15.2
4.5	23.3	9.4	25.3	41.5	11.1	49.4
6	22.7	12.9	24.9	39.6	16.6	47.8
7.5	22.6	11.4	25.4	39.1	14.2	49.8
9	23.4	10.0	24.5	41.8	12.1	46.1
10.5	23.0	10.0	23.6	40.6	12.0	42.7

**Table 3:** Inventories (B/m^2^) associated with all points collected at reference and study sites.

Reference site		Foot slope site 1		Terrace site 2	
Sample code	Inventory	Sample code	Inventory	Sample code	Inventory
R101	3804	PE101	2492	SD101	1278
R102	4086	PE102	2366	SD102	1328
R103	3543	PE103	2678	SD103	1374
R104	3511	PE104	2332	SD104	1239
R105	3564	PE105	1823	SD105	1289
R106	3675	PE106	1886	SD106	1303
R107	3790	PE107	2812	SD107	1232
R108	2965	PE108	2370	SD108	1264
R109	3800	PE109	1707	SD109	2617
R110	2864	PE110	2704	SD110	1217
R111	2791	PE111	1983	SD111	1846
R112	3003	PE112	2623	SD112	2345
R113	3250	PE113	2623	SD113	2481
R114	3069	PE114	2850	SD114	2167
R115	2979	PE115	2463	SD115	2296
R116	2944	PE116	2701	SD116	2420
R117	2499	PE117	2574	SD117	2428
R118	2840	PE118	2504	SD118	2478
R119	3108	PE119	2656	SD119	2242
R120	3135	PE120	2693	SD120	1057
R121	3616	PE121	2522	SD121	1092
R122	3014	PE122	2615	SD122	1050
R123	3369	PE123	2749	SD123	1128
R124	2927	PE124	2504	SD124	1210

## Data Availability

All data has been included.
